The article "Socioecological Challenges of Polio Supplementary Immunization Activities (SIAs) in the Asia-Pacific Region: A Systematic Review" was published in 2023. Journal: J Environ Public Health.

# Socioecological Challenges of Polio Supplementary Immunization Activities (SIAs) in the Asia-Pacific Region: A Systematic Review

**DOI:** 10.1155/2023/4801424

**Published:** 2023-01-28

**Authors:** Hanis Ahmad, Siti Aishah Sanef, Winda Zulaiha Shahabudin, Norfaqihah Mohtar, Mohd Rohaizat Hassan, Mohammad Saffree Jeffree, Khamisah Awang Lukman, Hasanain Faisal Ghazi, Syed Sharizman Syed Abdul Rahim

**Affiliations:** ^1^Department of Community Health, Faculty of Medicine, Universiti Kebangsaan Malaysia, Bandar Tun Razak, Kuala Lumpur, Malaysia; ^2^Borneo Medical and Health Research Centre, Faculty of Medicine and Health Sciences, Universiti Malaysia Sabah, Kota Kinabalu, Sabah, Malaysia; ^3^Department of Public Health Medicine, Faculty of Medicine and Health Sciences, Universiti Malaysia Sabah, Kota Kinabalu, Sabah, Malaysia; ^4^College of Nursing, Al-Bayan University, Baghdad, Iraq

## Abstract

**Background:**

Polio supplementary immunization activities (SIAs) are one of the polio eradication pillars in the Global Polio Eradication Initiative (GPEI) that increased the immunization coverage and made progress towards polio eradication. However, socioecological challenges faced during SIAs contribute to suboptimal campaign quality. The aim of this review is to identify the reported challenges during polio supplementary immunization activities (SIAs) and associated improvement strategies based on the socioecological model (SEM).

**Methods:**

Articles were searched from three databases which were WOS, Scopus, and PubMed. The systemic review identified the primary articles related to SIA that focused on the impact of immunization coverage, challenges, and improvement strategies. The inclusion criteria were open access English articles that were published between 2012 and 2021 and conducted in the Asia region.

**Results:**

There are nine articles described and explained regarding some form of supplementary immunization activities (SIAs) in their findings across Asia region. The majority of studies selected reported on post vaccination coverage and revealed a multifaceted challenge faced during SIAs which are widely diverse range from the microlevel of interpersonal aspects up to the macrolevel of government policy. Upon further analysis, the intervention at community level was the most dominant strategies reported during the SIA program.

**Conclusions:**

An effective SIAs program provides the opportunity to increase the national capacity of the polio immunization program, reducing inequities in service delivery and offering additional public health benefits in controlling polio outbreaks in both endemic and nonendemic countries. Strengthening routine immunization (RI) programmes is also important for the sustainability of SIA's programs. Despite the challenges and hurdles, many Asian countries exhibited great political willingness to boost polio immunization coverage through SIA efforts.

The article "Socioecological Challenges of Polio Supplementary Immunization Activities (SIAs) in the Asia-Pacific Region: A Systematic Review" was published in 2023. Journal: J Environ Public Health.

## 1. Introduction

Polio supplementary immunization activity (SIA) is a mass-immunization campaign that acts as supplementary immunization to complement routine immunization in order to achieve polio eradication [1]. It acts as one of the four main pillars of polio eradication in the Global Polio Eradication Initiative (GPEI) program, along with other pillars, namely, routine immunization, surveillance active for wild poliovirus, and targeted mop-up campaigns [1]. In general, SIA is implemented by international agencies such as the World Health Organization (WHO) and the United Nations Children's Fund (UNICEF) assisted by the local government, which is conducted at the national level during the National Immunization Days (NIDs) [2]. In a high-risk polio transmission area, SIAs are conducted during subnational immunization days (SNIDs) or through mop-up rounds following an outbreak of cases or through the outreach program and door-to-door campaigns in areas where routine immunization coverage is inadequate [2].

The main objective of SIA activities is to increase vaccine coverage by administering two doses with an interval of 4–6 weeks of oral polio vaccine to all children less than five years old, irrespective of their immunization status [1]. The nature of its activities enables to improve the accessibility of the marginalized populations to polio vaccination and overcome the vaccination seeking and awareness barriers in poor and difficult to reach populations [3]. Thus, it enhances protection towards susceptible age groups against polio and rapidly increases the immunity levels of general population, allowing to achieve herd immunity thresholds levels for polio and interrupt poliovirus chain transmission [1]. However, the massive use of oral polio vaccine (OPV) probably also results in the intensive secondary spread of shed vaccine virus among an underimmunized population [4].

Polio SIA has been implemented in western countries for the last 3 decades to improve polio vaccine coverage in lower average coverage regions. This effort proved to be effective as it showed more than a 30% increment in the polio vaccination coverage [5]. This good outcome of SIA was contributed by the broadening of vaccination health services and awareness especially among populations in limited access places [6, 7]. In Asian countries such as Indonesia, SIA seems able to reduce the poverty-related gap in getting the polio vaccine among the participants [8]. In the last two decades, about 10 billion polio vaccines have been successfully administered via SIA worldwide [9]. Despite demonstrations of SIA positive impacts, the challenges or barriers faced during conducting SIAs, particularly in limited resource countries, are rarely discussed.

The article "Socioecological Challenges of Polio Supplementary Immunization Activities (SIAs) in the Asia-Pacific Region: A Systematic Review" was published in 2023. Journal: J Environ Public Health.

Positive progress of GPEI reflects on declaration of free of poliovirus in 2014 from World Health Organization (WHO) South-East Asia Region and latest from WHO African Region in 2020 [2]. However, there are two countries that remain as polio endemic as Afghanistan and Pakistan. Even though the remaining endemic countries are only two, it has become a major concern especially among vulnerable countries with weak public health and travel or trade services due to the risk of importation of polio from endemic countries [1]. In addition to that, the risk of reintroduction of the virus can also happen in countries that have been cleared of the wild poliovirus but with low vaccination rates and inadequate and porous surveillance systems due to imported cases resulting from travel [10, 11]. Thus, GPEI had detailed this issue in the polio Eradication Strategy 2022–2026 to interrupt the poliovirus transmission in these two remaining polio endemic countries [3].

To achieve this objective, the gaps need to be comprehensively explored and intervene upon at each level of determinant factors, including challenges during implementing SIAs. Human and environmental factors can influence the acceptance of individuals towards SIA campaigns. According to Bronfenbrenner, individual development is shaped by human-environment interrelations. This socioecological model (SEM) demonstrates individual interests reflected by the interaction of one or more systems in the environment [12]. This theory has been adopted in a few studies, including public health related studies such as a study on factors related to immunization uptake [13–15]. With regard to health perspective, five multilevel factors from intrapersonal (individual characteristic and behaviour) [16], interpersonal (relationship between family and it social networks) [14], institutional (for example, health institution and its workers), community (for example, risk perception on vaccination uptake from community) [17], and policy (for example, providing role in delivering the healthcare access and services utilisation) [18] influence the population healthcare practice. Through reviewing polio SIA challenges by each of these levels interdependently, it enables to provide fundamental results that are useful for polio prevention plans that address the identified gaps from each level.

To the best of the authors' knowledge, there are no systematic reviews with contemporary evidence on the socioecological challenges and improvement strategies of polio SIA among middle-to-lower-income countries in the Asian region at this present time. Therefore, this systematic review aimed to identify the challenges of polio supplementary immunization activities (SIAs) based on the SEM approach in terms of intrapersonal, interpersonal, institutional, community, and policy together with the improvement strategies. The impact of SIAs in terms of immunization coverage was also summarised in this review.

The article "Socioecological Challenges of Polio Supplementary Immunization Activities (SIAs) in the Asia-Pacific Region: A Systematic Review" was published in 2023. Journal: J Environ Public Health.

## 2. Methods

### 2.1. Information Source

This systematic review method was guided by the Preferred Reporting Items for Systematic Reviews and Meta-Analyses (PRISMA) 2020 review protocol [19]. It targeted on articles that focused on the impact of the SIA activities in terms of immunization coverage, challenges, and improvement strategies. Related articles were searched from three databases (WOS, Scopus, and PubMed) from December 27^th^ 2021 until January 8^th^ 2022 by using keywords: polio, poliomyelitis, supplementary immunization activities (SIAs), mass-immunization campaigns, National Immunization Days (NIDs), immunization, and vaccination. The keywords were combined using advanced searching of field code (TITLE-ABS-KEY), phrase searching, truncation, and Boolean operators “OR” and “AND.”

### 2.2. Study Selection

The chosen primary articles were English language, open access, and published within 10 years (2012–2020) based on publication date. The inclusion criteria were

(1) Problem: challenges of polio SIA
(2) Interest:
  - Immunization coverage post SIA
  - SIA-related socioecological challenges are fully or partially focused on (i) intrapersonal or caregivers' factors, (ii) interpersonal between individual, social and peers, (iii) institutional from healthcare facilities and healthcare workers, (iv) community, and (v) policy in terms of immunization services and supply
  - Improvement strategies to overcome the SIA challenges
(3) Study type: empirical studies
(4) Context: Asia region

The exclusion criteria were

1. Not related to middle-income and lower-income countries
2. Case report or case series, technical notes, and modelling studies

During the selection process, two research team members searched for the relevant studies that met inclusion and exclusion criteria. Each of the 4 reviewers screened the titles and abstracts of all potential eligible articles. During the data confirmation process, full-text articles retrieved were randomly divided in two teams consisting of two members in each team. The two members in each team had screened the articles independently and reviewed the eligible articles interchangeably. Any disagreements were resolved by discussion and consensus between two members and in some instances with the input from the research team leader. The Mixed-Methods Appraisal Tool (MMAT) was used to evaluate the methodological quality of the finalised included studies before further data extraction and analyses were performed by the authors. The selection process followed the PRISMA flow diagram as shown in Figure 1.

The article "Socioecological Challenges of Polio Supplementary Immunization Activities (SIAs) in the Asia-Pacific Region: A Systematic Review" was published in 2023. Journal: J Environ Public Health.

The eligible articles were summarised in Excel form and categorised based on the outcome of interest, which were (i) immunization coverage status post SIA, (ii) challenges of SIA in terms of intrapersonal, interpersonal, institutional, community, and policy, and (iii) its improvement strategies.

## 3. Result

There are 33 full-text articles that fulfilled the inclusion criteria, but only nine (9) articles describe and explain some form of supplementary immunization activities (SIAs) in their findings around the Asia region. Based on Table 1, the studies mainly covered countries, namely, Pakistan, India, Bangladesh, Afghanistan, Malaysia, and Indonesia. In terms of study design selected for this review, the majority of the studies are observational studies, which out of total seven studies, it constitutes three quantitative descriptive studies, two qualitative studies, one nonrandomized study, and one mixed method study. Meanwhile, the rest are experimental studies, which are randomised control trials and quasi-experimental study.  Table 2 describes the articles included in the review based on the outcome measure, which mainly consists of vaccination coverage, barriers, and challenges, as well as the intervention strategies to SIA.

### 3.1. Vaccination Coverage

Upon further assessment, we discovered that five articles [1][3][4][6][8] answered the first research question, which was cited on the relation between the supplementary immunization activity (SIA) program and polio immunization coverage. Although the majority of studies [1][3][4][8] indicated a positive relationship between SIA campaigns and polio vaccination coverage, each study demonstrated the relationship in varying ways. Articles [1] and [8] indicated a significant increment of vaccination dose coverage with the integrated package of interventions. Meanwhile, article [3] showed a positive change in vaccination coverage that was substantially related to the number of SIA campaigns, while in articles [8], it was due to improved accessibility to SIA program via effective demographic and health surveillance. Despite these positive relations, insignificant change was also reported in article [6], where the primary outcome of this clinical trial which indicated no difference in vaccination coverage between the control and intervention groups who received community-level social mobilization initiative (CLSM).

The article "Socioecological Challenges of Polio Supplementary Immunization Activities (SIAs) in the Asia-Pacific Region: A Systematic Review" was published in 2023. Journal: J Environ Public Health.

### 3.2. Barrier or Challenges during the Supplementary Immunization Activities (SIAs)

Overall, the majority of articles selected for the final analysis constitute information regarding the barriers and challenges encountered during SIA programs. By referring to Bronfenbrenner's biological ecology system theory, the barriers and challenges reported in the selected articles shall be demonstrated in subcategory domains as follows: intrapersonal factor, interpersonal factor, institutional factor, community factor, and policy factor.

#### 3.2.1. Intrapersonal and Interpersonal

The intrapersonal and interpersonal challenges were solely reported in article [5], where the findings of this mixed-method study mainly constitute an overall negative perception toward the SIA program among surveyed parents. The quantitative part reported that among the 13% of respondents who did not participate in this SIAs, 73.9% refused to raise their hands due to fear of sterility, lack of faith in the polio vaccine, scepticism about the vaccination programs, and fear that the vaccine might contain religiously forbidden ingredients which were explained through the qualitative part of this study.

#### 3.2.2. Community

The challenges encountered at community level during the SIA program were solely reported in article [7], in which negative social behaviour toward the polio SIA program was found to be statistically significant with respect to the community's religion and educational background.

#### 3.2.3. Institutional

The institutional challenges during the SIA program were observed in articles [2][3] where both studies mainly touched on the weakness of the polio health surveillance and monitoring systems and the safety elements of healthcare workers, respectively. Article [2] showed that the data obtained from nonendemic middle-income and lower-income countries indicated no significant effect on the polio vaccination coverage despite the intense numbers of SIA programs as they were planned based on a poor polio health surveillance system. Other limitations were highlighted in article [3] which associated with the manually handling SIA monitoring process such as intensive resources, misreporting bias, and the risk of violence among healthcare workers. The workplace violence has been reported especially in places with poor security in which some of them have been assassinated.

#### 3.2.4. Government Policy

The challenge relates to the government policy mentioned in article [8], which reduced accessibility to routine vaccination services and SIA program among preschools and primary school students during the pandemic era due to movement control orders.

The article "Socioecological Challenges of Polio Supplementary Immunization Activities (SIAs) in the Asia-Pacific Region: A Systematic Review" was published in 2023. Journal: J Environ Public Health.

### 3.3. Intervention Strategy to Supplementary Immunization Activities (SIAs)

The following section will outline the intervention strategies reported in the selected articles. By referring to Bronfenbrenner's biological ecology system theory as well, the interventions strategy reported will be demonstrated in subcategory domains as in the previous barriers and challenges' part.

#### 3.3.1. Institutional

There are two studies [3][9] mentioned about the improvement strategies done in the healthcare system to enhance the function of the SIA program. Article [3] reported the introduction of short message service (SMS) via mobile phone to monitor the coverage of vaccination post SIA activities instead of a manual monitoring system. Whereas in article [9], the improvement done for healthcare workers through intervention package that includes SIA training, supervisions, and monitoring skills which has helped to improve the safety element during vaccination procedure and developed skills on risk assessment for SIA.

#### 3.3.2. Community

The majorities of articles [1][4][6][8] mentioned about the improvement strategies carried out at the community level. A positive outcome was reported in article [1], where the integration of community engagement into the polio SIA program showed a significant increment in immunization coverage while other articles focused more on explaining the different approaches utilized to achieve community engagement and mobilization. As in article [4], the desired SIA program's target is achieved through improved mapping of settlements wherein articles [6] and [8] highlighted that the appointment of a third person as a community representative that dedicating additional human resources and can help achieve desirable immunization outcomes in difficult-to-reach or programmatically challenged places. As mentioned in article [6], the third person plays a role in raising awareness about the SIA program among communities. Meanwhile, in article [8], it is mentioned that the selection of community mobilizers for the SIA program was among the community members from Community Health Volunteers (KOSPEN), health advisory panel, religious leaders, and goverment retirees.

#### 3.3.3. Government Policy

In article [8], the SIA program was done through smart partnership, utilizing multiple strategies that involved collaboration with other stakeholders such as the Ministry of Education and other entities.

## 4. Discussion

Strong routine immunization (RI) systems are important foundations for sustaining high levels of population immunity to vaccine-preventable diseases. Nonetheless, certain population groups continue to remain susceptible to vaccine-preventable diseases, either due to missing RI programmes or because of primary vaccination failures. Supplementary immunization activities (SIAs), also known as mass-immunization campaigns, were introduced as a proven strategy for increasing vaccination equity and rapidly increasing population immunity [28]. Therefore, in the present review, all observed evidence related to the impact, challenges, and improvement strategies of SIAs programs across the Asian region are summarized.

The article "Socioecological Challenges of Polio Supplementary Immunization Activities (SIAs) in the Asia-Pacific Region: A Systematic Review" was published in 2023. Journal: J Environ Public Health.

### 4.1. Impact of Routine Immunization following SIA Programs

The quality of the SIA is dependent on the impact of disease incidence assessed through disease surveillance. As a proxy for quality, polio SIAs should aim to achieve at least 95% coverage nationally to interrupt virus transmission (herd immunity). In this present systematic review, the evidence of polio SIA in strengthening the immunization coverage for polio routine immunization (RI) is summarized. The majority of the considered literature in the final analysis showed a positive increment of immunization coverage post SIA programs, except the finding seen in a quasi-experiment done in India in which the primary result showed no changes in immunization coverage following SIA activities [24]. The primary outcome for the present review study was consistent with a previous systematic review of 13 polio SIA studies across the African continents. The majority of these selected studies suggest a positive impact on polio vaccination coverage [29].

### 4.2. The Observed Challenges and Improved Strategies of Polio SIA

Over the last decade, the Global Polio Eradication Initiative (GPEI) has made steady progress on the path to eradication. In 2015 and 2019, wild poliovirus types 2 and 3 were declared eradicated, respectively. The final measures toward eradication, on the other hand, have proven to be the most challenging. The Polio Eradication Strategy 2022–2026 offers a comprehensive set of actions constituting of five strategic objectives, in which SIA programs are one of the solutions opted by public health specialists and other experts to mitigate the permanent eradication of polio infection. The majority of previous systemic reviews concentrate on the perceived benefits of the SIA program; they rarely discuss the challenges or improvement strategies. Therefore, this present systemic review study highlighted those aspects based on the social ecological model (SEM).

The reported barriers and challenges at the microlevel of socioecological strata are compromised of two important subcategorical domains, namely, intrapersonal and interpersonal factors. This present study indicates that parents' knowledge and attitudes toward SIA programs are poor in a polio endemic country, Pakistan. This is consistent with the findings of a similar study that investigated the knowledge and attitude of parents toward polio Routine Immunization (RI) programs done in Pakistan. Both studies highlighted the reasons for refusing polio vaccination; although the reasons for refusing vaccination are different to each other, they share one main reason due to false belief and lack of knowledge in polio vaccination effects. Despite the devastating outcome of polio infection, the majority of caretakers in Pakistan still have a negative attitude toward immunization; this is predictable as the majority of parent have a low level of knowledge regarding the benefits of polio immunization on their kid's health [30]. Another similar study was done in Nigeria; which has one of the highest vaccination refusal rate; they also perceived a similar finding where intrapersonal-interpersonal factors play an important role in determining caretaker personal attitude toward childhood vaccination program in general. This research suggests a significant relation between poor knowledge and refusal of immunization [31]. The relationship between knowledge and attitude of parents toward polio vaccination was clearly shown in that literature. This relation could not be generalised to other regions as the results were pooled from only a limited number of countries. Thus, advocation of studies from other high-risk countries is crucial to gain more evidence.

The article "Socioecological Challenges of Polio Supplementary Immunization Activities (SIAs) in the Asia-Pacific Region: A Systematic Review" was published in 2023. Journal: J Environ Public Health.

One of the strategic plans of the global polio elimination initiative (GPEI) is to generate vaccine acceptance by developing a better understanding of cultural and social barriers through social mobilization. Such intervention strategies at the community level were the most frequently observed findings reported in the selected articles. Many success stories can be found from studies included in this review, such as the two clinical trial studies conducted in Pakistan and India [20, 24]. These community intervention activities increased social and religious belief in the polio eradication mission by establishing a strong, positive relationship between community members and healthcare workers according to Choudhary et al. [24]. While another study done in Sabah, Malaysia, suggested that active participation of local influencers, such religious person, local leader, and retired government servants not only improved the social belief on the SIA activities but contributed to the success of the SIA program [26]. Although the detailed functions of community mobilizer in each article were not clearly mentioned, the following are some important targets to be achieved suggested by the GPEI, for example, shifting from a campaign-focused approach to instead making investments in sustained trust and relationship building with communities, reviewing accomplishments using the Minimum Quality Standards and Indicators for Community Engagement seeking opportunities for improving social mobilization activities in outbreak settings and including community engagement indicators in campaign preparedness dashboards to ensure social mobilization activities are tracked against meaningful indicators [1].

The article "Socioecological Challenges of Polio Supplementary Immunization Activities (SIAs) in the Asia-Pacific Region: A Systematic Review" was published in 2023. Journal: J Environ Public Health.

Detection of susceptible groups through a sensitive surveillance system is the most ultimate issue discussed under institutional factors in the selected articles in this review. It highlighted the limitations of the existing post SIA surveillance systems [21, 22]. In general, low-income countries are still utilizing manual surveillance systems which are found to have several limitations, for example, false reporting of immunization coverage. Manual surveillance also introduced extra usage of human, energy, and time resources. Without a good surveillance system, the targeted community (susceptible children) is overlooked from receiving OPV during the national mass-immunization campaigns. Therefore, some countries have shown no changes in immunization coverage despite numerous SIA activities due to poor polio surveillance systems. Thus, with the advancement of information technology, the utilisation of SMS is useful to replace the manual surveillance system in Pakistan [22]. As the use of SMS is considered less expensive compared to other virtual mediums, it is appropriate to be implemented in other regions with limited resources setting. This intervention can also be integrated into routine surveillance activity as mobile phone use is quite common nowadays [32]. Eventhough, none of the selected manuscripts in this present review report on the usage of web-based information and social networking during SIA among Asian countries, the usage was described among Western countries to overcome the vaccine hesitancy during the recent pandemic era by increasing knowledge. For example, in Italy, effective communication and health education on the importance of vaccines and their health were delivered to the general public through a web-based information platform [33]. Another example of reported intervention done at the institutional level was a modification of key activities indicators of the SIA program for healthcare workers in Nepal. It is comprised of the ultimate empowerment of SIA elements nationwide through training, social mobilization, supervision, and monitoring activities. Post training evolution showed a significant positive change in terms of knowledge of adverse events postimmunization [27].

The article "Socioecological Challenges of Polio Supplementary Immunization Activities (SIAs) in the Asia-Pacific Region: A Systematic Review" was published in 2023. Journal: J Environ Public Health.

In the modern era, a renewed focus on approaches to stakeholder engagement and political advocacy is a prerequisite to achieving eradication in both endemic and nonendemic countries through an effective mass vaccination campaign. However, the numbers of reported intervention strategies through such smart partnerships during SIAs program were extremely scarce in this present review. WHO and UNICEF recognised Malaysia efforts where the country demonstrated good collaboration during the SIA program by involving various stakeholders from both government and nongovernment agencies which boosted public confidence. A good cooperation system enables clear and effective communication between the District Health Office and the local authorities and other agencies. In certain countries, continuous conflict and insecurity may disrupt the campaigns due to restricted access in key geographical areas. Given the uncertainties around the ongoing subnational political situation, such collaboration has become one of the toughest hurdles to be adopted. In Pakistan, program success depends more on government political willingness or ownership of polio service delivery which requires systematic dialogue with the national and provincial leadership and other influential stakeholders. Good political willingness of polio vaccination program can be seen in Nigeria; after responding to insecurity and weakened health systems, Nigeria was eventually declared free of wild poliovirus case. The fundamental element in the success story was government commitment to regular review on progress of polio vaccination and good interconnection between federal and states level authorities. This also includes the country's commitment to fulfill financial resource requirement allocated under the Global Polio Elimination Initiative (GPEI) [1].

In cumulative, the reported findings in each selected article suggest that the challenges during the SIA program are widely diverse, ranging from the microlevel of interpersonal aspects up to the macrolevel of government policy. Advocating such an approach for synthesizing research evidence through social-ecological model (SEM) needs to be spotlighted in the future so that the improvement strategies can be carried out in the observed gaps area, which was previously left overlooked by the researchers. Failure to plan for an effective SIA that targets the susceptible groups reduces the chance of permanently interrupting all poliovirus transmission in endemic countries and increases the risk of outbreaks in nonendemic countries. Therefore, policymakers and healthcare providers can use the core information from our evidence summary to strengthen the existing policy and practice on polio supplementary immunization activities (SIAs), particularly during polio outbreaks. Although the discussion in the present study is concentrated on SIA-related issues back in the years before the pandemic, we are anticipating performing a systemic review that focuses on the post COVID-19 era in the future.

The article "Socioecological Challenges of Polio Supplementary Immunization Activities (SIAs) in the Asia-Pacific Region: A Systematic Review" was published in 2023. Journal: J Environ Public Health.

### 4.3. Strength and Limitations

To the best of our knowledge, this is the first preliminary systematic review ever conducted for the polio SIA program that focused on Asian countries. Previously, a few systemic reviews on polio mass-immunization campaigns have been conducted before, but none of those studies looked into the challenges and intervention strategies concurrently by adopting the socioecological model (SEM). Thus, the result of this present review shall yield a rigorous analysis of the challenges encountered during SIA from different countries' backgrounds. The use of SEM to present the subcategories domains for the reported intervention strategies is also considered superior to earlier studies as it shall identify any intervention gaps in each social-ecological level and will direct the policy makers or other authorities who involved in vaccination programs to set up a comprehensive approach in organizing SIA program especially during the polio outbreak. Nonetheless, there are some limitations encountered during the study's conduct that are mostly due to operational concerns. There is a possibility of publication bias attributable to endemic countries who have a greater ability to publish findings from polio SIAs than others, as this might limit the generalizability of results. An added limitation is that by focusing on the period from 2011 to 2013, we have missed several related studies that were conducted earlier. However, the focus was on extracting contemporary evidence to be adopted in future operational policies and practice in which the collected evidence enables the design of SIAs for all kinds of vaccine-immunize diseases.

## 5. Conclusion

The findings of this analysis reveal a multifaceted challenge faced during SIAs which are widely diverse, ranging from the microlevel of interpersonal aspects up to the macrolevel of government policy. By following the social-ecological model (SEM), the intervention strategic plan at each social hierarchy level must be incorporated into national and subnational vaccination strategic plans. An effective SIAs program provides the opportunity to increase the national capacity of polio immunization program, reducing inequities in service delivery and offering additional public health benefits in controlling polio outbreaks in both endemic and non-endemic countries. Strengthening RI programmes is also important for the sustainability of SIA's programs. Despite the challenges and hurdles, many Asian countries exhibited great political willingness to boost polio immunization coverage through SIA efforts.

The article "Socioecological Challenges of Polio Supplementary Immunization Activities (SIAs) in the Asia-Pacific Region: A Systematic Review" was published in 2023. Journal: J Environ Public Health.

## Figures and Tables

**Figure 1:** PRISMA flow diagram.

**Table 1:** Summary of study findings.

No.	Author (year), country	Title	Study design	Vaccination coverage	Challenges	Improvement strategies
1	Habib et al. (2017), Pakistan [20]	Community engagement and integrated health and polio immunization campaigns in conflict-affected areas of Pakistan: a cluster randomised controlled trial	Experimental (randomized control trial)	The estimated OPV coverage: before intervention (via routine vaccination: the coverage for children younger than 24 months of age was 43% in arm A, 52% arm B and 54% in arm C; post intervention: coverage was 75% in arm A compared with 82% in arm B and 84% in arm C significant increment in all arms with package of intervention	N/A	Arm A (control): intervention received the routine immunization and additional SIA. Arm B: received additional interventions with community outreach and mobilization using an enhanced communication package (community engagement) and provision of maternal and child. Health immunization services. Arm C: similar as above + IPV *∗*arm C shown greater increments after received combination of SIA + community outreach + IPV

2	Voorman and lyons (2016), LIC [21]	Measuring polio immunity to plan immunization activities	Observational	N/A	The numbers of SIA showed no effect on the dose coverage in several nonendemic MIC-LIC. Due to poor Polio surveillance system which used as surrogate indicators to determine the appropriate immunization activities as it done based on: (i) Caregiver self-report (ii) Lack of validated indicator (based on routine immunization)	N/A
3	Kazi et al. (2014), Pakistan [22]	Monitoring polio supplementary immunization activities using an automated short text messaging system in Karachi, Pakistan	Observational	Polio vaccination coverage reported as relationship between the numbers of campaigns per polio vaccination dose coverage	The monitoring system for SIA coverage done manually. Limitation: (i) Resource-intensive (ii) Utilizes convenience sampling and the 3rd party is prone to misreporting bias (iii) Exposes HCW to the risk of violence, especially in certain locations with poor security	Short message service (SMS) texts found to be an effective tool to measure the coverage of SIA activities in polio SIA in Karachi, Pakistan, showed that the coverages estimated using the SMS system were also like those recorded using lot QA sampling by WHO. For the monitoring of coverage in SIA, automated SMS-based systems appear to be an attractive and relatively inexpensive option

4	Helleringer et al. (2014), Indonesia, Bangladesh, Pakistan [8]	Polio supplementary immunization activities and equity in access to vaccination: evidence from the demographic and health surveys	Observational (cross sectional)	Indonesia 2007 (69.9%), Bangladesh 2011 (93.4%), Pakistan 2006 (81.9%).	N/A	To improve operational innovations in SIA implementation may have further improved the effectiveness of SIAs in reaching the poorest children, e.g., improved mapping of settlements and intensified activities of social mobilization and communication. Corroborate the idea that the SIA approach to health service delivery may be an important tool in promoting health equity

5	Khowaja et al. (2012), Pakistan [23]	Parental perceptions surrounding polio and self-reported nonparticipation in polio supplementary immunization activities in Karachi, Pakistan: a mixed methods study	Observational (mixed method study)	N/A	Quantitative 13% did not participate in one SIA: (i) 73.9% refused to participate (ii) 4.5% reported that the child was absent from home when the vaccinator visited (iii) 21.6% reported not having been contacted by a vaccinator qualitative (iv) Fear of sterility (v) Lack of faith in the polio vaccine (vi) Scepticism about the vaccination programme (vii) Fear that the vaccine might contain religiously forbidden ingredients	N/A
6	Choudhary et al. (2021), India [24]	Effectiveness of a community-level social mobilisation intervention in achieving the outcomes of polio vaccination campaigns during the post-polio-endemic period: evidence from CORE group polio project in Uttar Pradesh, India	Experimental (quasi-experimental)	SIA coverage post-polio-endemic period had insignificant change over time in both intervention group (community level social mobilisation) and nonintervention areas	Belief, fear	Vaccination campaign using community level social mobilisation

7	Podder et al. (2019), India [25]	Community perception toward intensified pulse polio immunization in post certification era: a mixed-method study in a high-risk area of Kolkata, West Bengal, India	Observational (cross-sectional)	N/A	Social behaviour is one of the barriers of polio SIA (IPPI-intensified pulse polio immunization) in Kolkata, West Bengal, India. It is statistically significant associated with respondent's attitude which directly link to gender, religion, and education. Result study showed the following: (i) Inadequate knowledge (32%) (ii) Unfavourable attitude (45%) (iii) Safety concern (5.7%) (iv) Spouse/elderly pressure (4.8%) (v) Sterility issues (1.9%) (vi) Hesitancy (16.2%)	N/A
8	Jiee et al. (2021), Malaysia [26]	Polio supplementary immunization activities during COVID-19 pandemic: experience from Penampang district, Sabah, Malaysia	Observational (case report)	OPV coverage has achieved more than 90% for both bOPV and mOPV	Movement control order enforcement causing the on-site activities involving the preschools and primary school student temporarily halted	Multiple vaccination strategies were utilized: static posts, mobile posts, house to house visits, school visits, mobile clinics and drive through. Schools' authorities were one of the most important partners in Polio SIAs since more than half of the targeted population were preschool and primary school children. Community health volunteers (KOSPEN), the health advisory panel, religious leaders, and government retirees were also involved as community mobilizers and recorder

9	Wallace et al. (2018), India [27]	Impact of an intervention to use a measles, rubella, and polio mass vaccination campaign to strengthen routine immunization services in Nepal	Experimental	N/A	N/A	Newly introduced or modified key activities in intervention package: SIA training, social mobilization, supervision, and monitoring were modified with RI messaging for healthcare providers from randomly selected 100 health care providers significant positive changes in terms of knowledge of adverse events post immunization (11% increase)

The article "Socioecological Challenges of Polio Supplementary Immunization Activities (SIAs) in the Asia-Pacific Region: A Systematic Review" was published in 2023. Journal: J Environ Public Health.

**Table 2:** Description of articles based on outcome measure.

Category	Subcategory	No. of studies	Article number^*∗*^
Vaccination coverage		6	[1][3][4][5][6][8]

Barrier or challenges in supplementary immunization activities (SIAs)	Intrapersonal	1	[5]
	Interpersonal	1	[5] [7]
	Institutional	2	[2][3]
	Community	N/A	—
	Policy	1	[8]

Intervention strategy to supplementary immunization activities (SIAs)	Intrapersonal	N/A	—
	Interpersonal	N/A	—
	Institutional	2	[3][9]
	Community	4	[1][4][6][8]
	Policy	1	[8]

^*∗*^The manuscripts (from 1 to 9 manuscripts) were numbered with the same numbering with which they are cited in Table 1.

## Data Availability

Data will only be provided upon request.
